The article "The Influence Mechanism of Knowledge Network Allocation Mechanism on Knowledge Distillation of High-Tech Enterprises" was published in 2022. Journal: Comput Intell Neurosci.

# The Influence Mechanism of Knowledge Network Allocation Mechanism on Knowledge Distillation of High-Tech Enterprises

**DOI:** 10.1155/2022/8246234

**Published:** 2022-04-25

**Authors:** Jianlin Yuan, Qilei Jiang, Yue Pan

**Affiliations:** College of Management, Liaoning University of Technology, Jinzhou 121001, China

## Abstract

Increasing global development competition highlights the value of knowledge innovation ability of high-tech enterprises. In order to acquire innovative knowledge, the mediating variables of knowledge field activity and knowledge stock ranking are selected; the moderating variables of knowledge resource pooling and knowledge evolution are adopted to construct the conceptual model and theoretical analysis framework of the influence mechanism of knowledge network arrangement mechanism on knowledge distillation; the moderating mediating effect model is derived; and the influence mechanism of knowledge network allocation mechanism on knowledge distillation of high-tech enterprises is clarified. 531 valid questionnaires were obtained online and offline, and non-percentile bootstrap based on deviation correction was used to empirically investigate the influence mechanism and transmission path of knowledge network allocation mechanism on knowledge distillation of high-tech enterprises. The empirical results show that the main effect of knowledge network pairing on knowledge distillation of high-tech enterprises is significant. The results show that knowledge field activity and knowledge stock ranking play a differential intermediary role in knowledge network allocation and knowledge distillation, knowledge field activity plays a partial intermediary role in knowledge network allocation and knowledge distillation, and knowledge stock ranking plays a partial intermediary role in knowledge network allocation and knowledge distillation. Pooling knowledge resources positively moderates the positive effect of knowledge network allocation mechanism on knowledge distillation and significantly positively moderates the mediating effect of knowledge field activity, and there is a moderated mediating effect derived from it. However, there is no significant moderating effect on knowledge stock ranking between knowledge network allocation mechanism and knowledge distillation. Knowledge evolution positively moderates the positive effect of knowledge network allocation mechanism on knowledge distillation, significantly positively moderates the mediating effect of knowledge field activity, and derives the moderated mediating effect. However, there is no significant moderating effect on knowledge stock ranking between knowledge network allocation mechanism and knowledge distillation. This paper makes an empirical study on the effect of knowledge allocation mechanism on knowledge distillation, enriches the connotation and application scope of knowledge distillation, defines the driving factors and formation mechanism of knowledge distillation, and further promotes the knowledge value and knowledge appreciation of high-tech enterprises. It has guiding and reference significance in the acquisition of innovation knowledge and the promotion of competitiveness of high-tech enterprises.

The article "The Influence Mechanism of Knowledge Network Allocation Mechanism on Knowledge Distillation of High-Tech Enterprises" was published in 2022. Journal: Comput Intell Neurosci.

## 1. Introduction

The 2020 epidemic has slowed down the development of the world economy, unilateralism has risen, and regaining the development of the world economy has become the main theme. Abandoning extensive development, advocating a refined pattern, and highlighting innovative economic drivers have become a new chapter in economic development. As a representative of innovation-driven development, high-tech enterprises rely on their unique industrial advantages for rapid knowledge spillover to help optimize and upgrade the industrial structure. With the rapid development of modern science and technology and the rapid expansion of knowledge, the ways for humans to obtain knowledge continue to expand. Networking and systemization have become an inevitable trend of knowledge utilization. However, the development of science and technology has also brought certain obstacles to the development of knowledge. With the rapid development of science and technology, the intensity and difficulty of knowledge and technology have increased gradually, and the redundancy of knowledge, the integration of knowledge, and the heterogeneity of knowledge have become effective knowledge. It is real dilemma of knowledge transformation. Wang believes that knowledge redundancy increases the cost of innovation-driven high-tech enterprises and highlights the obstacles to knowledge update [1]. The research results of Qin et al. show that knowledge integration seriously hinders knowledge innovation [2]. Malmström et al. believe that knowledge heterogeneity is a severe challenge faced by and delaying knowledge innovation [3]. It is of practical significance to overcome many obstacles in the process of knowledge innovation, improve the effectiveness and dimension of knowledge innovation, and drive high-tech enterprises to increase the economic contribution rate brought by innovation.

Take the knowledge network as the entry point; adopt the orderly allocation of knowledge; establish a scientific, reasonable, and orderly allocation mechanism; eliminate redundancy in knowledge transmission; reduce knowledge integration; assimilate knowledge heterogeneity; and accept effective knowledge content. This helps to improve the validity of knowledge and enhance the ability of knowledge innovation. The knowledge network breaks through the bottleneck of the continuous technological innovation of high-tech enterprises; gives full play to the characteristics of migration, iteration, and stability of the knowledge network; and leads the high-tech enterprises to start again. At present, knowledge network research is carried out around the three main characteristic dimensions of knowledge network structure, knowledge network relationship, and knowledge network subject. The research on the connection and density of the structural characteristics of the knowledge network reveals the validity and breadth of knowledge transfer and triggers the change of knowledge innovation capabilities. Dyer and Nobeoka's research on the tightness of structural connections between knowledge networks reveals that the transfer and transmission validity of tacit knowledge have a profound impact on the acceleration of knowledge flow and the conversion rate [4]. The characteristics of knowledge network relationship mainly focus on the influence of knowledge communication frequency, continuity, dependence, and other research knowledge on subject innovation. The characteristics of the main body of the knowledge network are based on the heterogeneity of the knowledge main body, including professional background, social status, and position difference, to study the validity of knowledge derivation. The heterogeneity of the subject of knowledge network is a “double-edged sword” for knowledge transfer and transformation. Effective knowledge exchange, communication, and integration between subjects are conducive to knowledge renewal, transformation, and iteration. On the contrary, it will seriously delay the transfer and exchange of knowledge. Knowledge update is stagnant, and the effectiveness of technological innovation is reduced. There are many research results of knowledge networks, which have greatly promoted knowledge innovation, but some content needs to be continuously deepened and extended. The knowledge network allocation mechanism can be the “golden key” of the research knowledge innovation highland, which can fully explore the transfer and transformation of knowledge. Validity promotes knowledge iteration and renewal, which is conducive to the transmission and diffusion of knowledge content. Knowledge distillation is the process of knowledge condensing. In the process of knowledge transfer, knowledge continues to iterate and sublimate. Knowledge distillation migrates the complex network to another simple and small network under the premise of ensuring the integrity of the value of knowledge as much as possible, so that the result of the lightweight analysis approximates the value obtained by the complex model. Knowledge distillation is a high degree of enrichment of the effectiveness of knowledge innovation, and it effectively promotes the formation of innovative power of high-tech enterprises.

The article "The Influence Mechanism of Knowledge Network Allocation Mechanism on Knowledge Distillation of High-Tech Enterprises" was published in 2022. Journal: Comput Intell Neurosci.

This article takes knowledge innovation as the main point and discusses the influence of knowledge network allocation mechanism on knowledge change and sublimation in the knowledge distillation of high-tech enterprises. The theoretical contribution mainly has three aspects: to enrich the content of related knowledge networks in the past, to further clarify the structural characteristics of knowledge networks, and to broaden the study of dependent variables before knowledge distillation. Secondly, it reveals the intermediary role of knowledge field activity and knowledge stock ranking between knowledge network allocation mechanism and knowledge distillation; again, it clarifies the regulation role of knowledge resource pooling and knowledge evolution in the activity of knowledge field and the ordering of knowledge stock on knowledge distillation. Finally, this research uses knowledge resource pooling and knowledge evolution to regulate the mediation model, expounds the influence of knowledge network allocation mechanism on knowledge distillation, and enriches the research results of knowledge network allocation mechanism on knowledge distillation. From a practical perspective, the research on the knowledge network allocation mechanism can have a profound impact on the knowledge innovation of high-tech enterprises. First of all, the knowledge network allocation mechanism has a good effect on knowledge distillation, which can help high-tech enterprises in knowledge innovation, enhance their competitiveness, and have a positive effect on high-tech enterprises' market development. Secondly, pay attention to the intermediary effect of knowledge field activity and knowledge stock ranking in the knowledge network allocation mechanism to knowledge distillation, and enhance the knowledge innovation ability of high-tech enterprises. Third, reconstruct the regulating effect of knowledge resource pooling and knowledge evolution on knowledge distillation in the activity of knowledge field, so as to continuously improve the knowledge innovation ability of high-tech enterprises. Finally, highlighting the role of knowledge resource pooling and knowledge evolution in the mediation of knowledge field activity on the corporate knowledge network allocation mechanism and knowledge distillation mediation can help the continuous flow and innovation of high-tech knowledge and enhance the competitiveness of high-tech enterprises.

The article "The Influence Mechanism of Knowledge Network Allocation Mechanism on Knowledge Distillation of High-Tech Enterprises" was published in 2022. Journal: Comput Intell Neurosci.

## 2. Related Literature Theories and Research Hypotheses

### 2.1. Knowledge Network Allocation Mechanism

Orchestration is derived from the vocabulary in music, and it means the orderly combination of related elements in music to present a beautiful and tactful musical effect, which highlights the harmony and coordination of musical elements. Orchestration emphasizes cooperation and innovation in the overall system and drives many scholars to pay attention to its application effects on the formation, stability, and evolution of the network. Li et al., Wang et al., Feller et al., and other scholars have empirically studied the causal relationship between network orchestration mechanism and network innovation and network cooperation [5–7]. Distribution effectively promotes the cross-organizational flow of knowledge and increases the value of knowledge exponentially. The effectiveness of the knowledge network allocation mechanism involves the process of effectively promoting the integration of knowledge network nodes and advancing the value of knowledge. The implementation of the knowledge network allocation process can effectively alleviate the technical, management, and organizational bottlenecks encountered by high-tech enterprises and realize the optimal allocation of various knowledge resources [8, 9].

The main core viewpoints in the theory of knowledge network allocation indicate that the core node is in the dominant position of the network. Through the effective combination, migration, and diffusion of knowledge resources, it completes the interaction between the members of the knowledge network and promotes the optimization of the combination and configuration of knowledge resources. High-tech enterprises bring the added value of knowledge. The core foundation of knowledge network allocation is knowledge resources. Through the integration and optimization of knowledge resources, the redundancy of knowledge is eliminated, the flexibility of knowledge strategy is enhanced, the fault tolerance in knowledge distillation is activated, and the stability of the knowledge network system is ensured. Dhanaraj and Parkhe define knowledge network allocation as a process of effectively integrating network knowledge resources through a series of purposeful behaviors, using scientific and reasonable technology, and exerting its best benefits [10]. High-tech enterprises implement and operate a knowledge network allocation mechanism to reduce the minimum redundancy of the authenticity of the knowledge system in the transmission of knowledge and promote the distillation of creative value of knowledge.

The article "The Influence Mechanism of Knowledge Network Allocation Mechanism on Knowledge Distillation of High-Tech Enterprises" was published in 2022. Journal: Comput Intell Neurosci.

According to the research results of Hurmelinna et al. and Feller et al., the knowledge network allocation mechanism includes knowledge transfer, knowledge iteration, and knowledge stability [7, 11].

The important value of high-tech enterprises is reflected in the resetting of knowledge value. In the process of knowledge transfer, integrating, optimizing, and reshaping of the original fragmented knowledge, maintaining knowledge flexibility, increasing knowledge toughness, weakening knowledge rigidity, and ultimately the authenticity of knowledge can be achieved the validity of knowledge can be enhanced through knowledge distillation. In the process of knowledge migration, integration, and optimization, knowledge iteration mainly focuses on the reorganization, deepening, and mining of knowledge on the basis of the original knowledge connotation, so as to fully display the excellent performance of knowledge in the new environment, eliminate the decaying dregs of knowledge, enhance the epidemic resistance of knowledge, improve the flexibility of knowledge, and weaken the rigidity of knowledge. The characteristics of knowledge (the fusion of tacit knowledge and explicit knowledge) increase the redundancy of knowledge in the process of knowledge transfer. Tacit knowledge refers to the characteristics of knowledge content that are difficult to accurately express. It is an inherent attribute of the knowledge growth process, which is mainly reflected in knowledge expressibility, implicitness, diversity, embeddedness, ambiguity, complexity, etc. The explicitness of knowledge is a manifestation of the externalization of the connotation of knowledge, which can directly act on the recipient and produce a certain effect. The knowledge network allocation mechanism fully excavates tacit knowledge, maintains knowledge flexibility to the greatest extent, and reduces knowledge redundancy. The flexibility of knowledge receptors also affects the validity of knowledge in the process of knowledge transfer. Knowledge distillation can ensure the integrity of knowledge, reduce the loss of knowledge in the process of knowledge transfer, and increase the fullness of knowledge.

Knowledge in the process of migration, integration, optimization and iteration focusing on the existing knowledge connotation, on the basis of knowledge restructuring, deepening, and mining, full display the knowledge in the new environment of excellent performance, excluding the rot meal of knowledge, enhance the knowledge of disease resistance, improve the knowledge of flexible, weakening the knowledge rigidity. The knowledge network allocation mechanism can establish a scientific and reasonable error correction mechanism based on the collaboration within the organization to increase the body's immunity within the knowledge network; moreover, through the interaction between the knowledge network system and external systems, it increases the overall adaptability of the knowledge network and improve knowledge purity and cleanliness of distillation. Knowledge iteration has undergone three changes, namely, knowledge capitalization, scenario-based, and ecologicalization. The capitalization of knowledge focuses on explicit knowledge, construction of knowledge content, and knowledge precipitation, to give full play to the value of knowledge and make it the intellectual asset of the organization. The contextualization of knowledge emphasizes people orientation emphasizes the integration and exchange of knowledge, pays attention to the construction of tacit knowledge such as skills and experience, and encourages the generation of knowledge connotation from work content. The ecologicalization of knowledge focuses on the construction of the knowledge ecosystem, emphasizes the diversity of knowledge formed by the realization of knowledge, fully taps the potential of knowledge, stimulates the inner driving force of knowledge, and promotes the upgrading of knowledge.

The article "The Influence Mechanism of Knowledge Network Allocation Mechanism on Knowledge Distillation of High-Tech Enterprises" was published in 2022. Journal: Comput Intell Neurosci.

Knowledge stability refers to the solidity of the overall knowledge structure and the integrity of knowledge content in the process of knowledge transfer and iteration. The incentives for knowledge stability mainly include three aspects, namely, the socialization of knowledge, the transformative nature of knowledge itself, and the inertia of knowledge. Social transformation, technological progress, social integration, knowledge diffusion, and convenience of knowledge dissemination methods threaten the stability of knowledge, constantly penetrating the inherent knowledge structure, changing the connotation of knowledge, and evolving knowledge. The knowledge network allocation mechanism can effectively adapt to changes in the external environment, effectively organize the integration of knowledge within the network, abandon the relevant inconsistent content within the knowledge network, and effectively transfer the essence of knowledge through knowledge distillation.

Aroles and Mclean believe that the relativity of knowledge stability is the prelude to the transformational transformation and is the result of the continuous coordination of internal and external environments [12]. It completes the differential integration of the body through the ontology structure and adsorption force and maintains the long-term innovation efficiency of the organization.

The article "The Influence Mechanism of Knowledge Network Allocation Mechanism on Knowledge Distillation of High-Tech Enterprises" was published in 2022. Journal: Comput Intell Neurosci.

Yu et al. pointed out that the stability of knowledge is greatly affected by the collaboration and psychological communication distance between subjects [13]. Das and Teng attributed knowledge stability to cooperation and competition, structural rigidity, and strategic flexibility [14]. Ernst and Bamford proved that the rigidity of knowledge structure is the deep root cause of knowledge instability [15].

The research results of Wang and You show that if the frequency of communication between organizations and the transparency of communication content are increased, the effect and speed of knowledge transfer can be improved; in addition, the exchange of explicit knowledge between organizations, salary adjustments, and organizational learning ability can help improve the quality and stability of knowledge [16].

Through case studies, Gill and Butler believe that the key factors affecting knowledge stability include cooperation trust, knowledge-gene conflict, and knowledge-gene stickiness [17]. Among them, cooperative trust can promote the evolution of knowledge based on the basic form of the knowledge structure, while genetic conflict and genetic stickiness pose challenges to the stable structure of knowledge. Within the knowledge network, the key resources possessed by the knowledge ontology, the knowledge subject's attitude towards knowledge transfer, and the behavior of individual knowledge can all constrain the effect of knowledge transfer within the knowledge network and affect the stability of knowledge.

Based on the above research, this article proposes hypotheses:

  Hypothesis 1: The knowledge network allocation mechanism has a positive effect on knowledge distillation.
  Hypothesis 1.1: Knowledge transfer has a positive effect on knowledge distillation.
  Hypothesis 1.2: Knowledge iteration has a positive effect on knowledge distillation.
  Hypothesis 1.3: Knowledge stability has a positive effect on knowledge distillation.

### 2.2. The Intermediary Effect of Knowledge Field Activity and Knowledge Stock Ranking

Through the electromagnetic field theory in physics, Japanese scholars Nonaka and Takeuchi took the lead in defining the connotation of the knowledge field, which refers to the spatial pattern formed in the process of knowledge transfer, knowledge diffusion, and knowledge differentiation [18]. In this space, subjects interact with each other. In this space, each subject interacts, influences, constantly running-in, embeds, and rebirths with each other, and the value of knowledge is sublimated. Based on the different ways of knowledge transformation within the enterprise, the knowledge field is mainly divided into initiation, system, dialogue, and practice. The knowledge field is divided into two types: strong and weak. If the members in the knowledge field have close bonds, strong node signals, and high frequency of mutual interaction, it is a strong knowledge field; otherwise, it is a weak knowledge field. Based on the concept of knowledge field, scholars derived the concept of knowledge field activity from the perspective of its dynamic activity; that is, the subjective values of knowledge exchange and communication are the same, the willingness to share knowledge is strong, and knowledge interaction and communication can proceed with sincerity. Gan and Qi draw on Li Ling's research results and believe that the activity of the knowledge field can be divided into the activity and openness of the knowledge field [19]. Combining the relevant research results of knowledge field at home and abroad, it is believed that the activity of knowledge field has the attribute of dual structure. The activity of the knowledge field is affected by the collision, friction, and mutual reorganization between the internal subjects, and the external environment can also stimulate and determine the activity and the openness of the knowledge field.

The article "The Influence Mechanism of Knowledge Network Allocation Mechanism on Knowledge Distillation of High-Tech Enterprises" was published in 2022. Journal: Comput Intell Neurosci.

In the knowledge network system, the optimization, combination, and allocation of knowledge resources among members can promote the continuous improvement of the knowledge stock level of each member in the knowledge space. Nell et al. believe that the difference in the internal structure of the knowledge field leads to the hierarchical difference between the knowledge stocks among the members of the knowledge field, and the different rankings of the knowledge resource stocks within the knowledge field cause the imbalance of the knowledge stock [20]. Many scholars have studied the characteristics of the distribution of knowledge stock among different subjects within the knowledge network system and paid attention to the rules presented by the order of the knowledge stock among the members of the knowledge field. Ciabuschi et al. believed that due to the different internal structure of the knowledge field, the sorting of knowledge stocks showed a binary complex of complex and simple attributes [21]. They were inspired by the knowledge of series and parallel circuits in physics and believed that the sorting of knowledge stocks the concept can also be divided into serial sorting of knowledge stock and parallel sorting of knowledge stock. Majchrzak et al. showed that the study believes that the parallel sorting of knowledge stock includes knowledge exclusivity and knowledge configuration [22]. The parallel sorting of knowledge stock is mainly reflected in the integration and application of knowledge components, while the nature of the knowledge stock owned by the enterprise itself has no essential change. Wang believes that the serialization of knowledge stock is the iterative connection of knowledge based on coupling and embedding of knowledge resources to form a new body of knowledge, which is the embodiment of knowledge modularity [23]. The complexity of the knowledge network system increases the difficulty of knowledge identification, nesting, and migration. With the help of AI, it can perceive the activity of the knowledge field; scientifically and rationally sort the knowledge stock; and solve the series of problems of knowledge transfer, knowledge iteration, and knowledge stability in the knowledge network arrangement.

The article "The Influence Mechanism of Knowledge Network Allocation Mechanism on Knowledge Distillation of High-Tech Enterprises" was published in 2022. Journal: Comput Intell Neurosci.

Under the knowledge network allocation mechanism, knowledge distillation is mainly realized through the following two intermediary mechanisms: “knowledge field activity” and “knowledge stock ranking.” First, under the action of the knowledge network allocation mechanism, excellent knowledge genes can be preserved, promote the activity of the knowledge field, increase the activity of the knowledge field, enhance knowledge flexibility and knowledge resilience, highlight the power of knowledge dissemination and the degree of knowledge diffusion, and fully represent knowledge. Dynamic nature drives knowledge to display its content in a new posture, stimulates the matching and strategy between internal structure and external demand changes, better expresses the inherent attributes of knowledge, and realizes the essence of enterprise knowledge distillation. Second, the knowledge network orchestration mechanism derived needs further expression of knowledge and knowledge essence, sort through stock of knowledge, a clear knowledge of regularity and precision of the knowledge essence, led the overall knowledge structure stability, displayed the scientific thinking and the development of the context of the location and structure more clear can guide. On a certain basis, it strengthens the characteristics of independent learning and intelligent development of knowledge. To sum up, “knowledge field activity” and “knowledge stock ranking” play a certain intermediary role in the influencing process of knowledge network allocation mechanism on knowledge distillation. The following hypotheses are put forward:

  Hypothesis 2: The activity of the knowledge field plays an intermediary role in the process of the positive influence of the knowledge network allocation mechanism on the knowledge distillation.
  Hypothesis 3: The ranking of knowledge stock plays an intermediary role in the process of the positive influence of the knowledge network allocation mechanism on knowledge distillation.

The article "The Influence Mechanism of Knowledge Network Allocation Mechanism on Knowledge Distillation of High-Tech Enterprises" was published in 2022. Journal: Comput Intell Neurosci.

### 2.3. Knowledge Resource Pooling and the Moderating Effect of Knowledge Evolution

#### 2.3.1. Knowledge Resource Pooling

The knowledge resource pool is a metaphor borrowed from the physical form of the pool. The process of resource pooling is to integrate resources to a certain extent and satisfy their needs in the form, method, and content that satisfy customers. The knowledge resource pool has knowledge resource storage control, load balancing, resource quantity control, resource restoration, orderly arrangement of resources, etc. The primary function of the knowledge resource pool is the storage and control of knowledge, which gathers the knowledge resources possessed by the enterprise, and this kind of agglomeration is orderly and not disorderly. Knowledge resource pooling has the functions of storing knowledge, effectively increasing the knowledge stock, improving the efficiency of knowledge updating, ranking the knowledge stock to ensure the orderly utilization of knowledge resources, and speeding up the knowledge distillation of high-tech enterprises. Knowledge resource pooling has two obvious characteristics: precipitation and reorganization. The pooling and precipitation function of knowledge resources refer to the action of the knowledge ontology to further enrich and enhance the connotation according to the external environment. Knowledge achieves the purpose of strengthening the bones and muscles through knowledge pooling, knowledge itself is upgraded, the activity of knowledge is enhanced, and the active ability of knowledge field is further displayed. The heavy function of knowledge resource pooling refers to the increase in the amount of knowledge accumulation, the targeted discrimination and selection of knowledge, the reloading of similar and dissimilar knowledge elements, the update and superposition of knowledge content, and the expansion of knowledge connotation. Breaking through the limitations of original knowledge, knowledge activity has been effectively improved.

With the help of the pooling technology of image data collection, the concept of knowledge pooling is introduced. Knowledge pooling refers to the use of minimal and simple knowledge connotation to express the essential knowledge of the objective subject, thereby forming knowledge integration and generalization. Knowledge resource pooling has the functions of knowledge coupling, aggregation, and collaboration. Knowledge resource pooling is the process of resource standardization. In extension, knowledge resources eliminate the wrong, incorrect, and decayed content of the knowledge content through the precipitation, purification, catalysis, and reaction of knowledge and sublimate the purity of the knowledge content. Knowledge resource pooling can promote the activity and flexibility of knowledge, and strengthen the resilience of the knowledge network. Through the precipitation of time, the knowledge resource pool reduces the stickiness of knowledge, increases the combination of knowledge, and highlights the integration of knowledge, so that knowledge can be reorganized and evolved according to needs. The knowledge resource pool emphasizes the filtering, precipitation, and combination functions of the knowledge resource pool. After knowledge resources are screened, filtered, and precipitated, the cleanliness, flexibility, and combination of knowledge are improved, and the excellent knowledge genes can be inherited, reorganized, and sublimated. The extraction can be completed, the activity of the knowledge field is further enhanced, the stock of knowledge continues to increase, and the distillation of knowledge can be brought into play.

The article "The Influence Mechanism of Knowledge Network Allocation Mechanism on Knowledge Distillation of High-Tech Enterprises" was published in 2022. Journal: Comput Intell Neurosci.

#### 2.3.2. Knowledge Evolution

Borrowing from Darwin's theory of evolution, introducing the theory of evolution of knowledge, knowledge is adapted to the process experienced by the new essence through the steps of precipitation, evolution, and catalysis. The theory of evolution is based on the survival of the fittest, and the evolution of knowledge emphasizes the degree of matching and coordination with the environment. Ding and Wu believe that knowledge is a kind of hypothesis, which survives continuous struggle and is a competitive result [24]. In practice, through trial and error, the incorrect knowledge content is corrected, and the knowledge content that does not meet external needs is eliminated.

Knowledge evolution has dual attributes. The content structure of knowledge determines its development endurance, and the external environment of knowledge promotes internal knowledge. Connelly et al. emphasize the robustness of the internal structure of knowledge evolution and believe that knowledge continuously strengthens its own semantic structure, strengthens its muscles, is rich in content, adapts to changes in the external environment, promotes the transformation and upgrading of knowledge itself, and adapts to new concepts of knowledge [25]. The essence of the content is preserved, highlighting the internal robustness of knowledge. Xu and Wang believe that excellent knowledge genes have a keen sense of the external environment, actively perceive changes, carry out self-change, and inherit the excellent connotation of knowledge resources [26]. In the evolution of knowledge, changes in the external environment act on the internal structure of knowledge to generate mutations in the knowledge genes and be passed on. Fang et al. emphasized that the external environment has the function of knowledge evolution, and the stable internal structure and sensitive perception of knowledge promote the internal adjustment of the knowledge body, adapt to the changes in the external environment, enhance the knowledge connotation, and continue excellent genetic knowledge [27]. Aiming at the three biological evolutionary mechanisms of mutation, heredity, and natural selection, Xu and Wang divided knowledge evolution into three different paths: convergent evolution, divergent evolution, and coevolution [26]. Changes in the external environment (such as changes in competitors, adjustments in national policies, and technological innovations) break the original knowledge structure, recombine the internal genes of knowledge, reshape it into new knowledge connotations, enhance the activity of the knowledge field, strengthen the knowledge stock, and make knowledge present a clear structural feature of errors, which promotes the realization of knowledge distillation. Although the formation of knowledge expression is different, the value added to the subject of knowledge is equivalent; that is, knowledge converges and evolves. Knowledge assimilation strengthens and extends the knowledge bones and the knowledge connotation can be sublimated, and the role of knowledge distillation is obvious. The knowledge subject generated from the same traceability, due to changes in the external environment (such as cultural differences, different concepts, and different social customs), has not been changed much, significant changes have taken place in the substantive connotation of the knowledge subject, and it is already on a development track that does not intersect, which is the divergent evolution of knowledge. The difference of knowledge evolution brings the variability characteristics of the activity of the knowledge field and the heterogeneity of knowledge stock and highlights the reproducibility of knowledge, the continuous evolution and breakthrough of the essence of knowledge, and the acceleration of knowledge distillation. Coevolution means that the internal structure of knowledge adapts to changes in the external environment, produces internal reorganization of knowledge, and produces new knowledge essentials, so that the overall internal structure of knowledge does not restructure, but it satisfies the requirements of the external environment well.

The article "The Influence Mechanism of Knowledge Network Allocation Mechanism on Knowledge Distillation of High-Tech Enterprises" was published in 2022. Journal: Comput Intell Neurosci.

The improvement and upgrading of the knowledge distillation function of high-tech enterprises will further enhance the competitiveness of high-tech enterprises and promote the efficiency of knowledge transformation. In the process of knowledge distillation of high-tech enterprises, knowledge resource pooling and knowledge evolution strengthen the process of knowledge distillation by adjusting the activity of the knowledge field and the ranking of knowledge stocks. The activity of knowledge field and the sorting of knowledge stock through knowledge resource pooling and knowledge evolution are mainly manifested in two mechanisms for the regulation of knowledge distillation. First, the knowledge resource pooling has contributed to the precipitation, extraction, and differentiation of knowledge. This strengthens the characteristics of knowledge connotation; increases the flexibility, cohesion, and cleanliness of knowledge; and further highlights the activity of knowledge. Furthermore, the aggregation of knowledge fields increases, and the stock of knowledge continues to accumulate. The hierarchical structure of knowledge is becoming more and more obvious, and the coupling effect of knowledge resources further promotes the highly condensed knowledge content, forms the agglomeration of knowledge connotation, and demonstrates the flexibility and resilience of knowledge. Under the regulation of the pooling of knowledge resources, the degree of knowledge integration is further improved. Sublimation enhances the stability of the knowledge network, the efficiency of the knowledge network is continuously improved, the knowledge diffusion power is enhanced, and the patency of the knowledge distillation function is improved. Second, knowledge evolution further promotes the convergence and differentiation of knowledge, strengthens the unity and homogeneity of knowledge, sublimates knowledge activity, and continuously improves the stock of knowledge. Knowledge evolution further promotes the ability of knowledge to adapt to changes in the external environment. According to the needs of objective subjects, the connotation of knowledge is adjusted, the integration efficiency of knowledge content is promoted, and the distillation of knowledge is adjusted. From the above analysis, this article believes that knowledge resource pooling and knowledge evolution play a moderating role in the activity of knowledge field, the ranking of knowledge stock, and the distillation of enterprise knowledge.

Based on the above analysis, the following hypotheses are proposed:

  Hypothesis 4: The knowledge resource pool positively regulates the influence of knowledge field activity and knowledge stock ranking on knowledge distillation; that is, the higher the level of knowledge resource pool, the stronger the influence of knowledge field activity and knowledge stock ranking on knowledge distillation.
  Hypothesis 5: Knowledge evolution positively regulates the influence of knowledge field activity and knowledge stock ranking on knowledge distillation; that is, the higher the level of knowledge evolution, the stronger the influence of knowledge field activity and knowledge stock ranking on knowledge distillation.

The article "The Influence Mechanism of Knowledge Network Allocation Mechanism on Knowledge Distillation of High-Tech Enterprises" was published in 2022. Journal: Comput Intell Neurosci.

### 2.4. Regulated Mediation

Hypothesis 2 explained the mediating effect of knowledge field activity, and hypothesis 4 explained the regulating effect of knowledge resource pooling on the relationship between knowledge field activity and knowledge distillation. Combining these two aspects, this study further infers that knowledge resource pooling is in the compilation of knowledge networks. The allocation mechanism plays a regulatory role in the entire mediation mechanism process of knowledge distillation through the activity of the knowledge field, forming a regulated mediation role; that is, the knowledge resource pooling helps the knowledge network allocation mechanism to actively transform the knowledge distillation into knowledge distillation through the activity of the knowledge field. Specifically, with the enhancement of the knowledge resource pooling function, the speed and accuracy of knowledge transfer between organizations can be continuously improved. The knowledge network allocation mechanism provides more internal and external opportunities, facilities, and platforms for the knowledge field activity, so it can facilitate the inoculation and evolution of the iterative and updating of knowledge system and improve the value performance of knowledge distillation. Conversely, knowledge resource pooling is at a low level, and the efficiency of internal and external knowledge integration slows down. Even if the knowledge network orchestration drives the active operation mechanism and operation mode of the knowledge field, the enterprise knowledge organization system will still lack effective operation control. Knowledge resource pooling is unable to promote continuous knowledge innovation and reduce the efficiency of knowledge distillation.

Hypothesis 2 illustrates the mediating role of knowledge field activity, and hypothesis 5 illustrates the mediating role of knowledge evolution in the relationship between knowledge field activity and knowledge distillation. Combining these two aspects, this study further infers the mechanism of knowledge evolution in the knowledge network allocation mechanism. The activity of the knowledge field plays a regulatory role in the entire intermediary mechanism of knowledge distillation, forming a regulated intermediary effect; that is, knowledge evolution contributes to the active transformation of the knowledge network orchestration mechanism to knowledge distillation through the activity of the knowledge field. Specifically, with the improvement of the function of knowledge evolution, the maturity of the interorganizational knowledge system has been further strengthened, and the sense of knowledge has been improved, which facilitates the proactive knowledge exchange with the external environment, improves the efficiency of knowledge change, enhances the flexibility of organizational knowledge, and realizes the smooth development of knowledge distillation. Conversely, knowledge evolution is not active enough, the inherent initiative of knowledge genes cannot be effectively stimulated, and the update efficiency of knowledge connotation slows down. Even if the knowledge network orchestration drives the inherent initiative of the activity of the knowledge field, the operating efficiency of the enterprise knowledge organization system cannot be effective. The improvement cannot continue to promote knowledge innovation and reduce the efficiency of knowledge distillation. Based on the above analysis, this study believes that knowledge resource pooling and knowledge evolution have a certain moderating effect on the mediating effect of knowledge field activity on knowledge network allocation and knowledge distillation, and the following hypotheses are put forward accordingly.

  Hypothesis 6: Knowledge resource pool and knowledge evolution positively regulate the knowledge network allocation to influence the mediating effect of knowledge distillation through the activity of knowledge field; that is, the higher the level of knowledge resource pool and knowledge evolution, the stronger the mediating effect of knowledge field activity.
  Hypothesis 7: Knowledge resource pool and knowledge evolution are positively regulated. Knowledge network allocation affects the mediating effect of knowledge distillation through the ranking of knowledge stock; that is, the higher the level of knowledge resource pool and knowledge evolution, the stronger the mediating effect of knowledge stock ranking.

The article "The Influence Mechanism of Knowledge Network Allocation Mechanism on Knowledge Distillation of High-Tech Enterprises" was published in 2022. Journal: Comput Intell Neurosci.

Based on the above analysis, this research believes that the knowledge network allocation mechanism in high-tech enterprises can promote knowledge distillation. At the same time, knowledge network allocation mechanism further promotes enterprise knowledge distillation and reduces organizational knowledge consumption through mediation of knowledge field activity and knowledge stock ranking. The mediating role of inventory ranking further promotes enterprise knowledge distillation and reduces organizational knowledge loss. Knowledge resource pooling and knowledge evolution, respectively, play a regulatory role in the activity of knowledge fields and the relationship between knowledge inventory ranking and knowledge distillation. Forming a regulated mediation role can adjust the intermediary media in a targeted manner, promote the integration of enterprise knowledge, and ensure the resilience of enterprise knowledge update and the flexibility of knowledge iteration. Based on this, this article constructs a theoretical conceptual model and overall theoretical analysis framework for the relationship between enterprise knowledge network allocation mechanism, knowledge field activity, knowledge stock ranking, knowledge resource pooling, knowledge evolution, and knowledge distillation and discusses the knowledge network allocation mechanism in depth. The internal influence mechanism and transmission path of knowledge distillation of high-tech enterprises are shown in Figure 1.

## 3. Research Design

### 3.1. Data Sources

This article takes employees of high-tech enterprises as the survey objects. The sample data comes from more than a dozen regions in the eastern provinces. It mainly uses online and offline data survey methods. Online questionnaire surveys mainly send questionnaires to obtain research-related data; offline questionnaire surveys are mainly conducted online, using the questionnaire star as a platform to obtain relevant survey data. The industry to which the enterprise belongs is the eastern high-tech enterprise. In order to obtain accurate survey data and avoid the psychological suggestion effect caused by the relevant items of the questionnaire on the survey subjects, the questionnaire is protected; at the same time, in order to ensure the accuracy of the questionnaire data, the respondents are anonymous and confidential before the survey is done. In this survey, a total of 552 questionnaires were issued, 542 were recovered, 11 questionnaires were removed, and 531 questionnaires were valid, with an effective rate of 97.79%. The characteristics of the sample are described in Table 1.

### 3.2. Selection and Measurement of Variables

The scale used in the problem analysis mainly comes from the mature scale design at home and abroad. The variable measurement adopts the 7-point Likert scale system. 1 to 7, respectively, represent, “completely disagree” to “completely agree.” The specific measurement indicators and basis are shown in Table 2.

## 4. Empirical Result Analysis

### 4.1. Descriptive Statistical Analysis

The relevant variables in the conceptual model and theoretical analysis framework are described, and the results are shown in Table 3. The Pearson correlation coefficients of different variables are between 0.5 and 0.7, indicating that the variables have a certain correlation.

The article "The Influence Mechanism of Knowledge Network Allocation Mechanism on Knowledge Distillation of High-Tech Enterprises" was published in 2022. Journal: Comput Intell Neurosci.

### 4.2. Reliability and Validity Test of Scale

This article adopts the method of controlling nonmeasurable potential factors to test the common method deviation phenomenon involved in this article. The new latent label variable is set as the knowledge filter. Compared with the goodness-of-fit index corresponding to the structural equation model before control, the goodness-of-fit index of the structural equation model after control and the main goodness-of-fit index are both relatively poor. The amount of change is as follows: the absolute change corresponding to the ratio between the chi-square and the degree of freedom is 0.094, the absolute change of the NFI indicator is 0.03, the absolute change of the IFI indicator is 0.03, the absolute change of the CFI indicator is 0.03, and the absolute change of the RMSEA indicator is 0.02, which further shows that there is no serious common variance bias in this paper.

The variable reliability and validity test results (as shown in Table 4) show that it has good credibility (Cronbach's > 0.7). The structural framework of each variable is excellent (KMO test values are all >0.5). The variable combination reliability value (CR > 0.70) indicates that the variable has good construction reliability. The variable AVE value (AV > 0.750) indicates that the variable convergent validity is better.

### 4.3. Conceptual Model and Research Hypothesis Testing

#### 4.3.1. The Main Effect Analysis and Test of the Allocation Mechanism of Knowledge Network

According to the main effect test results of the knowledge network allocation mechanism in Table 5, the regression coefficient *β* of knowledge distillation is 0.6343, the *p* test value is not greater than 0.05, and the lower and upper limits of the regression coefficient interval estimation are 0.5224 and 0.7463, respectively, and it shows that the knowledge network allocation mechanism has a significant positive promotion on knowledge distillation. The knowledge network allocation mechanism can enhance the order of knowledge, strengthen the coupling and optimization of knowledge genes, and promote the knowledge distillation of high-tech enterprises.

#### 4.3.2. Analysis and Test of the Mediating Effect of Knowledge Field Activity

Drawing lessons from Wen et al.'s idea and process of intermediary effect testing, using the bootstrap method in the Process plug-in to analyze and test the intermediary effect of knowledge field activity, we present the results in Table 6 [43].

The article "The Influence Mechanism of Knowledge Network Allocation Mechanism on Knowledge Distillation of High-Tech Enterprises" was published in 2022. Journal: Comput Intell Neurosci.

The mediating role of knowledge field activity is tested by a three-step method.

Firstly, we test the influence of the knowledge network allocation mechanism on the activity of the knowledge field. According to Model 1 in Table 6, it can be seen that the knowledge network allocation mechanism has a significant positive effect on the activity of the knowledge field (*β* = 0.7905, *p* < 0.05). Secondly, Model 2 shows the degree of influence of knowledge network allocation mechanism on knowledge distillation. Knowledge network organization has a significant positive effect on knowledge distillation (*β* = 0.6343, *p* < 0.05). Finally, Model 3 adds knowledge field activity to the regression model. Comparing the results of Model 2 and Model 3, we find that the influence of knowledge network composition on knowledge distillation is reduced, from *β* = 0.6343 (*p* < 0.05) to *β* = 0.1723 (*p* < 0.05) and the activity of the knowledge field has a significant partial mediating effect.  Table 7 clearly shows the mediating role of knowledge field activity. The knowledge network orchestration mechanism can have a positive effect on knowledge distillation through knowledge field activity.

#### 4.3.3. Analysis and Examination of the Mediation Effect of Knowledge Stock Ranking

Drawing lessons from Wen et al.'s idea and process of intermediary effect testing, using the bootstrap method in the Process plug-in to analyze and test the intermediary effect of knowledge stock sorting, we provide the results in Table 8 [43].

The mediating role of the knowledge stock ranking is tested by a three-step method.

First, the impact of knowledge network allocation and knowledge inventory ranking is tested. According to Table 8, Model 1 knowledge network allocation mechanism has a significant positive impact on knowledge inventory ranking (*β* = 0.8144, *p* < 0.05). Second, Model 2 shows the degree of influence of the knowledge network allocation mechanism on knowledge distillation, and the knowledge network allocation mechanism has a significant positive effect on knowledge distillation (*β* = 0.6343, *p* < 0.05). Finally, Model 3 puts the ranking of knowledge stock into the regression model for analysis. Comparing Model 2 and Model 3, we find that the influence of knowledge network compilation on knowledge distillation decreases to a higher degree and from a higher level *β* = 0.8925 (*p* < 0.05). To the lower level *β* = 0.5925 (*p* < 0.05), the sorting of knowledge stock has a significant partial mediating effect.  Table 9 clearly shows the mediating effect of the ranking of the knowledge stock, and the knowledge network orchestration mechanism can have a positive effect on the knowledge distillation through the ranking of the knowledge stock.

The article "The Influence Mechanism of Knowledge Network Allocation Mechanism on Knowledge Distillation of High-Tech Enterprises" was published in 2022. Journal: Comput Intell Neurosci.

#### 4.3.4. Analysis and Examination of the Moderating Effect of Knowledge Resource Pooling

We draw lessons from Wen et al.'s thought and process of regulating effect test and use the bootstrap method in the Process plug-in to complete the analysis and test of the regulating effect of knowledge resource pooling (Table 10) [44]. According to Model 1 in Table 10, knowledge field activity and knowledge resource pooling have a significant positive impact on knowledge distillation (*β* = 0.2541, *p* < 0.05; *β* = 0.4475, *p* < 0.05), and the interaction effect between the two is obvious (*β* = 0.1518, *p* < 0.05), indicating that knowledge resource pooling can have a better moderating effect between knowledge field activity and knowledge distillation.  Table 11 further describes the effect of knowledge resource pooling on the relationship between knowledge field activity and knowledge distillation in different situations and promotes the improvement of enterprise innovation capabilities. Model 2 shows that the ranking of knowledge stock and the pooling of knowledge resources have a significant positive impact on knowledge distillation (*β* = 0.0817, *p* < 0.05; *β* = 0.8837, *p* < 0.05), but the interaction effect is not significant. Knowledge resource pooling is no obvious moderating effect between the inventory ranking and the knowledge distillation (*β* = 0.0066, *p* > 0.05; the confidence interval contains 0).

#### 4.3.5. Analysis and Examination of the Moderating Effect of Knowledge Evolution

We draw lessons from Wen et al.'s thought and process of regulating effect testing and use the bootstrap method in the Process plug-in to complete the analysis and testing of the regulating effect of knowledge evolution (Table 12) [44]. According to Model 1 in Table 12, it can be seen that knowledge field activity and knowledge evolution have a significant positive impact on knowledge distillation (*β* = 0.1465, *P* < 0.05; *β* = 0.5970, *p* < 0.05) and the interaction effect between the two is obvious (*β* = 0.0923, *p* < 0.05), indicating that knowledge evolution can have a better moderating effect on the relationship between knowledge field activity and knowledge distillation.  Table 13 further describes the effect of knowledge evolution on the relationship between knowledge field activity and knowledge distillation in different situations and promotes the improvement of enterprise innovation capabilities. Model 2 shows that the ranking of knowledge stock and knowledge evolution have a significant positive impact on knowledge distillation (*β* = 0.8858, *p* < 0.05; *β* = 0.1159, *p* < 0.05) but the interaction effect is not significant. Knowledge evolution is no obvious moderating effect between the distillation relationships. There is no obvious moderating effect between the distillation relationships (*β* = 0.0062, *p* > 0.05; the confidence interval contains 0).

The article "The Influence Mechanism of Knowledge Network Allocation Mechanism on Knowledge Distillation of High-Tech Enterprises" was published in 2022. Journal: Comput Intell Neurosci.

#### 4.3.6. Analysis and Examination of Mediated Mediation

With the help of the bootstrap method in the Process plug-in, the adjusted mediation effect is tested. According to the results of Model 1 in Table 14, the interaction product term of knowledge field activity and knowledge resource pooling is significant (0.1120, *p* < 0.05), indicating that the mediating effect of knowledge field activity is regulated by knowledge resource pooling, which positively affects knowledge distillation.  Table 15 shows that when knowledge resource pooling is high (one standard deviation above the mean), the mediation value of knowledge network allocation mechanism through knowledge field activity to knowledge distillation is 0.0671, and the 95% bias-corrected bootstrap confidence interval is [ 0.0390, 0.1711]; excluding 0, the mediating effect is significant. When knowledge resource pooling is low (one standard deviation below the mean), the mediating effect of knowledge network allocation mechanism through knowledge field activity to knowledge distillation is 0.0390. The 95% deviation-corrected Bootstrap confidence interval is [0. 0252, 0.1120], excluding 0, the mediating effect is significant; the mediating indirect effect value is very different between the high level and low level of the knowledge resource pooling (*p* < 0.05, CI [0.0170, 0.0747]). It shows that when the pooling of knowledge resources becomes stronger, the activity of the knowledge field will significantly increase the mediating effect between the knowledge allocation mechanism and the knowledge distillation (Table 16).

With the help of the bootstrap method in the Process plug-in, the test of the adjusted mediation is completed. According to Model 2 in Table 14, the interaction product term of knowledge field activity and knowledge evolution is significant (0.1187, *p* < 0.05), indicating that the mediating role of knowledge field activity is regulated by knowledge evolution and positively affects knowledge distillation. When the level of knowledge evolution is high (one standard deviation above the mean), the mediation value of the knowledge network allocation mechanism through the activity of the knowledge field to the knowledge distillation is 0.1003, and the 95% deviation correction confidence interval is [0.0380, 0.1589]. Including 0, the mediating effect is significant. When the level of knowledge evolution is low (one standard deviation below the mean), the mediation value of the knowledge network allocation mechanism through the activity of the knowledge field to the knowledge distillation is 0.0618, and the 95% deviation correction confidence interval is [0.0315, 0.1280]. Excluding 0, the mediating effect is significant. There is a significant difference between the mediating indirect effect value when the knowledge evolution is high and the mediating indirect effect value when the knowledge evolution is low (*p* < 0.05, CI [0 0122, 0.0727]). It shows that when knowledge evolves more intensely, the mediating effect of knowledge field activity between knowledge allocation mechanism and knowledge distillation is significantly enhanced.

The article "The Influence Mechanism of Knowledge Network Allocation Mechanism on Knowledge Distillation of High-Tech Enterprises" was published in 2022. Journal: Comput Intell Neurosci.

## 5. Conclusion and Discussion

### 5.1. Analysis Conclusion

Based on the perspective of knowledge innovation theory, this paper takes the activity of knowledge field and the ranking of knowledge stock as intermediary variables and explores the influence mechanism and transmission path of knowledge network allocation mechanism on the knowledge distillation of high-tech enterprises under the effect of the adjustment of knowledge resource pooling and knowledge evolution. The following empirical results are obtained:

1. The knowledge network allocation mechanism has a significant positive impact on the knowledge distillation of high-tech enterprises. High-tech enterprises should continuously update and iterate knowledge to ensure the smooth operation of their knowledge system and knowledge structure. After high-tech enterprises have sufficient intellectual capital, knowledge, and technology, they not only need to attract more alliance enterprises to participate in the cooperation network. In order to promote the continuous expansion of their own knowledge stock, they also should actively seek new partners; increase their own competitive advantage, leadership, and influence in the industry; constantly transfer, update, and iterate knowledge; and promote the continuous growth and change of their own knowledge.
2. The activity of the knowledge field and the ranking of the knowledge stock play a part of the intermediary role in the relationship between the allocation mechanism of the long-term knowledge network of high-tech enterprises and the knowledge distillation.
3. Knowledge resource pooling and knowledge evolution have a positive regulating effect between the activity of the knowledge field of high-tech enterprises and the distillation of knowledge. The external environment of the enterprise is relatively stable. The enterprise can make full use of its own advantages to accumulate and replace knowledge, complete its updating, and share it with partners in appropriate ways. The integration internal and external environment knowledge of enterprises can further promote the iterative upgrading of knowledge and information sources between enterprises and partners and further promote the efficiency of knowledge transfer.
4. The active mediation of knowledge field is regulated by knowledge resource pooling and knowledge evolution, and there is a significant positive influence between knowledge network allocation and knowledge distillation. The mediating role of knowledge inventory ranking is regulated by knowledge resource pooling and knowledge evolution, and the positive influence between knowledge network allocation and knowledge distillation is not significant. It has provided assistance to the innovation ability of high-tech enterprises.

The article "The Influence Mechanism of Knowledge Network Allocation Mechanism on Knowledge Distillation of High-Tech Enterprises" was published in 2022. Journal: Comput Intell Neurosci.

### 5.2. Theoretical Meaning

1. This article expands the research on the antecedent variables of knowledge distillation.
2. In the past, the research on the antecedent variables of knowledge distillation focused on the expression of information, proposing that the acquisition of high-value knowledge information from the massive information on the network has relatively little impact on the information in the network. Through the research of this article, the influence mechanism of knowledge distillation information transmission has been further enriched, and the related research of knowledge distillation has been expanded.
3. This research hints at the mediating role of knowledge field activity and knowledge stock ranking between knowledge network arrangement and knowledge distillation.
4. Under the knowledge network allocation mechanism, the paper focuses on the action mechanism of knowledge field activity and knowledge stock ranking on the knowledge innovation ability of high-tech enterprises, that is, the paper riches the content about the research of the tacit knowledge and explicit knowledge, which further activates the research that knowledge field activity and knowledge stock ranking influence knowledge renewal, migration, and iteration of high-tech enterprises. It enriches the action mechanism of knowledge field activity and knowledge stock ranking on knowledge renewal of high-tech enterprises.
5. This research clarifies the regulation function of knowledge resource pooling and knowledge evolution in the activity of knowledge field and the ranking of knowledge stock on knowledge distillation through knowledge resource pooling and knowledge evolution. Knowledge resource pooling and knowledge evolution are introduced as the moderating variables to further explain the regulation effect of high-tech enterprise knowledge resource pooling and knowledge evolution on the activity of knowledge field and the ordering of knowledge stock on knowledge distillation, revealing the inherent logical relationship of knowledge transfer and launching an in-depth interpretation and analysis of it.
6. This research uses knowledge resource pooling and knowledge evolution to regulate the mediation model, expounds the influence of knowledge network allocation mechanism on knowledge distillation, enriches the research results of knowledge network allocation mechanism on knowledge distillation, and further expounds the mechanism of knowledge resource pooling and knowledge evolution on the mediating role of knowledge evolution in knowledge network allocation mechanism on knowledge distillation.

The article "The Influence Mechanism of Knowledge Network Allocation Mechanism on Knowledge Distillation of High-Tech Enterprises" was published in 2022. Journal: Comput Intell Neurosci.

### 5.3. Practical Significance

The research conclusions of this article have certain reference value for management practice; they are specifically manifested in the following.

First of all, the knowledge network allocation mechanism has a good effect on knowledge distillation, which can help high-tech enterprises in knowledge innovation, enhance their competitiveness, and have a positive effect on high-tech enterprises' market development. The knowledge network allocation mechanism provides organizations with advanced concepts of integration and optimization of internal and external knowledge, technology, patents, etc.; promotes the establishment of innovative mechanisms for enterprises; exerts the initiative of knowledge subjects; and continuously promotes knowledge distillation and knowledge renewal.

Secondly, pay attention to the intermediary effect of knowledge field activity and knowledge stock ranking in the knowledge network allocation mechanism to knowledge distillation, and enhance the knowledge innovation ability of high-tech enterprises. The activity of the knowledge field enhances knowledge openness and communication efficiency, guarantees the upgrading and iteration of the knowledge content of high-tech enterprises, integrates the knowledge structure of high-tech enterprises, and strengthens the innovation driving force of high-tech enterprises. The ranking of knowledge stock can guide the direction of knowledge accumulation of high-tech enterprise employees, stimulate the internal knowledge acquisition ability of employees, promote the transfer and exchange of knowledge within the enterprise, enhance the cohesion of high-tech knowledge, strengthen the bones and muscles, and achieve the connotation of high-tech knowledge sublimation.

Thirdly, reconstruct the regulating effect of knowledge resource pooling and knowledge evolution on knowledge distillation in the activity of knowledge field. Through research, knowledge resource pooling and knowledge evolution play a regulatory role in the activity of knowledge field and knowledge distillation. High-tech enterprises can use this as a breakthrough point to strengthen knowledge precipitation, accelerate the circulation process of knowledge, and give play to the openness of knowledge field activity. Improve the sublimation mechanism of high-tech enterprises' knowledge, and promote the ability of knowledge innovation.

The article "The Influence Mechanism of Knowledge Network Allocation Mechanism on Knowledge Distillation of High-Tech Enterprises" was published in 2022. Journal: Comput Intell Neurosci.

Finally, the research highlights the mediating function of knowledge resource pooling and knowledge evolution in the activity of knowledge field to the mediation mechanism of enterprise knowledge network integration and knowledge distillation. Knowledge resource pooling and knowledge evolution play a regulated function in the intermediary effect of knowledge field activity on the enterprise knowledge network allocation mechanism and knowledge distillation.

### 5.4. Research Limitations and Prospects

Although the research conclusions of this paper have certain theoretical value and practical significance for the construction of enterprise knowledge innovation mechanism, there are still some shortcomings.

First of all, the data used in this article comes from questionnaires. When the respondents fill out the questionnaires, the subjective preferences of the technicians are unavoidable. In the future, interviews and surveys can be adopted to verify the data so as to improve the accuracy of the sample data. At the same time, the longitudinal data can be also collected and summarized according to different time points, so as to obtain a more accurate causal relationship path. In addition, according to the different logical relations between variables, in future research, different analysis software can be used to study the influence mechanism of the knowledge network allocation mechanism.

Secondly, in the construction of the knowledge network allocation mechanism to the knowledge distillation model, the selection of the intermediary variable and the moderating variable and the influence mechanism need to be further deepened. The selection of intermediary variables and moderating variables refers to the research purpose of this article and the research of related scholars, but it should be fully explored in the elaboration, in order to deepen the research on the mechanism of knowledge network allocation and the principle of knowledge distillation.

## Figures and Tables

**Figure 1:** Research conceptual model diagram.

**Table 1:** Sample feature description.

	Attributes	Quantity/proportion
Area	Eastern region	531
Attribution level	State-owned and state-controlled	15
	Joint venture and private	26
Industry	High-tech industry	41
Years of establishment	Less than 5 years	17
	5–10 years	16
	More than 10 years	8
Enterprise size	300 people or less	134
	300–1000 people	286
	More than 1000 people	111
Respondent's position	Senior technical staff	45.2%
	Midlevel technical staff	54.8%
Respondent's education	Undergraduate	275
	Bachelor degree and above	256
Working years under investigation	Less than 5 years	138
	5–10 years	247
	More than 10 years	146
Surveyed gender	Male	282 people
	Female	249 people

The article "The Influence Mechanism of Knowledge Network Allocation Mechanism on Knowledge Distillation of High-Tech Enterprises" was published in 2022. Journal: Comput Intell Neurosci.

**Table 2:** Measurement indicators and basis.

Variable	Dimension	Item	References
Knowledge network allocation mechanism	Knowledge transferability	Paying attention to the dynamic learning of new knowledge by employees	Dhanaraj and Parkhe, Hurmelinna et al. [10, 11]
		Number of patents owned by the company	
		Channels for corporate employees to communicate	
		Organizational learning ability	
	Knowledge iteration	Frequency of employees going out	Eisingerich et al., Leischnig et al., Bi et al. [28–30]
		Having a good cooperative relationship with external companies	
		Enterprise technology development process	
	Knowledge stability	Diversification of corporate knowledge sources	
		Product development cycle	
		Enterprise technology update cycle	
Knowledge field activity	Knowledge coordination	The mobility of enterprise technical staff	Senoo et al., Ding [31, 32]
		The difference of enterprise technical personnel	
	Knowledge exchange	Differences in organizational systems	
	Knowledge learning	Responsibility with partners	Prabhu et al., Wu and Shanley, Liu and Zhou [33–35]^.^
Knowledge inventory ranking	Technological innovation	There is good cohesion among employees within the enterprise	Chen et al., Gao and Liu, etc. [36, 37]
		Smooth corporate interaction and communication	
		Strong active learning atmosphere	
		Enterprise personnel participating in external technical exchanges and cooperation	
	Funding	The enterprise's ability to update and adjust the knowledge stock according to the changes in the external environment of the enterprise in a timely manner	Connelly and Zweig, Liden et al. [25, 38].
Knowledge resource pooling	Organization cooperation	The talents owned by the enterprise having rich knowledge and experience	
		The company actively encouraging internal members to organize various learning, communication, and discussion activities	
Knowledge evolution	Brand recognition	The company's relatively complete and reasonable distribution of key knowledge	
		Number of enterprise high-tech reserves	Kang and Liu [39]
Knowledge distillation		Enterprise R&D investment amount	Hu et al., Pan et al., etc. [40–42]
		Continuous R&D span in a certain field	
		Enterprise's ability to acquire external knowledge	
		The enterprise having the knowledge to meet the needs of the enterprise and society	
		Enterprise high-tech transformation	
		Business and local cooperation	
		Corporate brand being recognized by the society	
		Conversion and utilization efficiency of enterprise scientific research funds	
		Enterprise technology being recognized in the industry	
		Flexibility of enterprise organization	

The article "The Influence Mechanism of Knowledge Network Allocation Mechanism on Knowledge Distillation of High-Tech Enterprises" was published in 2022. Journal: Comput Intell Neurosci.

**Table 3:** Descriptive statistics and correlation coefficients.

	Average value	Standard deviation	B1	B2	B3	B4	B5	B6	B7
Knowledge transferability	3.7056	1.16454	1.000						
Knowledge iteration	3.3070	1.05820	0.607^*∗∗*^	1.000					
Knowledge stability	3.4937	0.98213	0.633^*∗∗*^	0.659^*∗∗*^	1.000				
Knowledge field activity	3.2395	1.04810	0.604^*∗∗*^	0.577^*∗∗*^	0.646^*∗∗*^	1.000			
Knowledge inventory ranking	3.3140	0.95400	0.594^*∗∗*^	0.556^*∗∗*^	0.622^*∗∗*^	0.558^*∗∗*^	1.000		
Knowledge resource pooling	3.2453	1.39234	0.549^*∗∗*^	0.516^*∗∗*^	0.501^*∗∗*^	0.587^*∗∗*^	0.548^*∗∗*^	1.000	
Knowledge evolution	3.4928	1.39427	0.614^*∗∗*^	0.576^*∗∗*^	0.621^*∗∗*^	0.631^*∗∗*^	0.666^*∗∗*^	0.671^*∗∗*^	1.000
Knowledge distillation	3.2916	1.34221	0.634^*∗∗*^	0.547^*∗∗*^	0.603^*∗∗*^	0.575^*∗∗*^	0.614^*∗∗*^	0.593^*∗∗*^	0.632^*∗∗*^

*Note.* ^*∗∗*^Significant at the 5% level.

**Table 4:** Reliability and validity test of the scale.

	Number of items	KMO test value	Cronbach's coefficient	Factor loading factor	CR	AVE
Knowledge transfer	4	0.540	0.722	0.808	0.8273	0.5465
				0.776		
				0.700		
				0.664		

Knowledge iteration	5	0.640	0.657	0.428	0.8322	0.5121
				0.587		
				0.740		
				0.845		
				0.878		

Knowledge stability	5	0.677	0.756	0.441	0.8369	0.5273
				0.456		
				0.806		
				0.904		
				0.876		

Knowledge field activity	4	0.556	0.643	0.299	0.7960	0.5299
				0.553		
				0.941		
				0.916		

Knowledge inventory ranking	5	0.719	0.600	0.012	0.7724	0.5065
				0.137		
				0.879		
				0.938		
				0.928		

Knowledge resource pooling	3	0.688	0.788	0.789	0.8763	0.7029
				0.864		
				0.860		

Knowledge evolution	3	0.740	0.892	0.900	0.9328	0.8222
				0.895		
				0.925		

Knowledge distillation	4	0.721	0.7422	0.763	0.8386	0.7525
				0.815		
				0.673		
				0.752		

**Table 5:** The main effect test results of the knowledge network allocation mechanism.

Main effect	Effect	se	*t*	*p*	LLCI	ULCI
Knowledge network orchestration	0.6343	0.0570	11.1336	0.0000	0.5224	0.7463

**Table 6:** Active mediation of knowledge field.

	Model 1	Model 2	Model 3
	Dependent variable knowledge field activity	Dependent variable knowledge distillation	Dependent variable knowledge distillation
Knowledge network orchestration	0.7905^*∗∗∗*^ (*t* = 21.8989) (0.7196, 0.8614)	0.6343^*∗∗∗*^ (*t* = 11.1336) (0.5224, 0.7463)	0.5821^*∗∗∗*^ (*t* = 10.1284) (0.5137, 0.7541)
Knowledge field activity			0.1723^*∗∗∗*^ (*t* = 3.4148) (0.0732, 0.2714)

*Note.* ^*∗∗∗*^Significant at the 1% level.

The article "The Influence Mechanism of Knowledge Network Allocation Mechanism on Knowledge Distillation of High-Tech Enterprises" was published in 2022. Journal: Comput Intell Neurosci.

**Table 7:** The mediating effect and confidence interval of knowledge field activity.

	Indirect effect estimation	95% confidence interval	
	(standardization)	Lower limit	Upper limit
Knowledge field activity	0.1262	0.0527	0.2120

**Table 8:** Test results of the mediation effect of the ranking of the stock of knowledge.

	Model 1	Model 2	Model 3
	Dependent variable knowledge inventory ranking	Dependent variable knowledge distillation	Dependent variable knowledge distillation
Knowledge network orchestration	0.8144^*∗∗∗*^ (*t* = 22.4844) (0.7432, 0.8855)	0.6343^*∗∗∗*^ (*t* = 11.1336) (0.5224, 0.7463)	0.5925^*∗∗∗*^ (*t* = 12.1526) (0.5135, 0.7662)
Knowledge inventory ranking			0.0361^*∗∗∗*^ (*t* = 0.2932) (0.0840, 0.2258)

*Note.* ^*∗∗∗*^Significant at the 1% level.

**Table 9:** The mediation effect and confidence interval of the ranking of knowledge stock.

	Indirect effect estimation	95% confidence interval	
	(standardization)	Lower limit	Upper limit
Knowledge inventory ranking	0.1362	0.0471	0.2238

**Table 10:** The adjustment effect of knowledge resource pooling.

	Model 1	Model 2
	Dependent variable knowledge distillation	Dependent variable knowledge distillation
*Intermediary*		
Knowledge field activity	0.2541^*∗∗∗*^ (*t* = 5.9322) (0.1699, 0.3382)	
Knowledge inventory ranking		0.0817^*∗∗∗*^ (*t* = 5.1393) (0.0593, 0.1327)

*Moderator*		
Knowledge resource pooling	0.4475^*∗∗∗*^ (*t* = 10.4503) (0.3634, 0.5316)	0.8837^*∗∗∗*^ (*t* = 47.2774) (0.8470, 0.9205)
Interactive product term		
Knowledge field activity *∗* knowledge resource pooling	0.1518^*∗∗∗*^ (*t* = 4.9562) (0.0916, 0.2120)	
Knowledge inventory ranking *∗* knowledge resource pooling		0.0066 (*t* = 0.4639) (−0.0214, 0.0346)

*Note.* ^*∗∗∗*^Significant at the 1% level.

**Table 11:** Confidence interval of the moderating effect of knowledge resource pooling.

Adjusting the intensity	Effect estimate (standardization)	95% confidence interval	
		Lower limit	Upper limit
High	0.3898^*∗∗∗*^ (*t* = 8.3922)	0.2986	0.4811
Middle	0.2808^*∗∗∗*^ (*t* = 6.6571)	0.1979	0.3637
Low	0.0628^*∗∗∗*^ (*t* = 3.0019)	0.0603	0.1859

*Note.* ^*∗∗∗*^Significant at the 1% level.

**Table 12:** Test results of the regulation of knowledge evolution.

	Model 1	Model 2
	Dependent variable knowledge distillation	Dependent variable knowledge distillation
*Intermediary*		
Knowledge field activity	0.1465^*∗∗∗*^ (*t* = 3.5585) (0.0656, 0.2274)	
Knowledge inventory ranking		0.8588^*∗∗∗*^ (*t* = 41.5985) (0.8183, 0.8994)

*Moderator*		
Knowledge evolution	0.5970^*∗∗∗*^ (*t* = 14.5540) (0.5164, 0.6776)	0.1159^*∗∗∗*^ (*t* = 5.6261) (0.0754, 0.1564)

*Interactive product term*		
Knowledge field activity*∗*knowledge evolution	0.0923^*∗∗∗*^ (*t* = 3.3399) (0.0380, 0.1465)	
Knowledge inventory ranking*∗*knowledge evolution		0.0062 (*t* = 0.4358) (−0.0216, 0.0339)

*Note.* ^*∗∗∗*^Significant at the 1% level.

The article "The Influence Mechanism of Knowledge Network Allocation Mechanism on Knowledge Distillation of High-Tech Enterprises" was published in 2022. Journal: Comput Intell Neurosci.

**Table 13:** Knowledge evolution regulation and confidence interval.

Adjusting the intensity	Effect estimate (standardization)	95% confidence interval	
		Lower limit	Upper limit
High	0.2453^*∗∗∗*^ (*t* = 5.1524)	0.1518	0.3389
Middle	0.1348^*∗∗∗*^ (*t* = 3.2280)	0.0528	0.2168
Low	0.0468^*∗∗∗*^ (*t* = 2.0538)	0.0589	0.1525

*Note.* ^*∗∗∗*^Significant at the 1% level.

**Table 14:** Test results of regulated mediation.

	Model 1	Model 2	Model 3	Model 4
	Dependent variable knowledge distillation	Dependent variable knowledge field activity	Dependent variable knowledge distillation	Dependent variable knowledge field activity
*Independent variable*				
Knowledge network allocation mechanism	0.5291^*∗∗∗*^ (*t* = 10.2451) (0.4357, 0.6225)	0.5257^*∗∗∗*^ (*t* = 13.8668) (0.4512, 0.6002)	0.6251^*∗∗∗*^ (*t* = 11.1238) (0.5224, 0.7463)	0.4994^*∗∗∗*^ (*t* = 11.9502) (0.4173, 0.5816)

*Mediating variable*				
Knowledge field activity	0.1623^*∗∗∗*^ (*t* = 3.4148) (0.0689, 0.2556)		0.1723^*∗∗∗*^ (*t* = 3.5618) (0.9732, 0.2714)	

*Moderator*				
Knowledge resource pooling		0.2901^*∗∗∗*^ (*t* = 7.5683) (0.2148, 0.3654)		
Knowledge evolution				0.3003^*∗∗∗*^ (*t* = 7.1507) (0.2178, 0.3828)

*Interactive product term*				
Knowledge field activity *∗* knowledge resource pooling		0.1120^*∗∗∗*^ (*t* = 4.4282) (0.0623, 0.1616)		
Knowledge field activity*∗*knowledge evolution				0.1187^*∗∗∗*^ (*t* = 4.7884) (0.0700, 0.1674)

*Note.* ^*∗∗∗*^Significant at the 1% level.

**Table 15:** The adjusted mediation test results estimated by the non-percentile bootstrap method based on bias correction (knowledge network allocation⟶knowledge field activity⟶knowledge resource pooling⟶knowledge distillation).

Regulating variable action intensity	Indirect effect (standardization)	95% confidence interval	
		Lower limit	Upper limit
High (+IS.D)	0.0671	0.0390	0.1711
Low (−IS.D)	0.0390	0.0252	0.1120
Difference between high and low	0.0363	0.0170	0.0747

**Table 16:** The adjusted mediation effect estimated by the non-percentile bootstrap method based on bias correction and its test results (knowledge network allocation mechanism⟶knowledge field activity⟶knowledge evolution⟶knowledge distillation).

Regulating variable action intensity	Indirect effect (standardization)	95% confidence interval	
		Lower limit	Upper limit
High (+IS.D)	0.1003	0.0380	0.1589
Low (−IS.D)	0.0618	0.0315	0.1280
Difference between high and low	0.0385	0.0122	0.0727

The article "The Influence Mechanism of Knowledge Network Allocation Mechanism on Knowledge Distillation of High-Tech Enterprises" was published in 2022. Journal: Comput Intell Neurosci.

## Data Availability

The data used to support the findings of this study are available from the corresponding author upon request.
